# Oncolytic Virotherapies and Adjuvant Gut Microbiome Therapeutics to Enhance Efficacy Against Malignant Gliomas

**DOI:** 10.3390/v16111775

**Published:** 2024-11-14

**Authors:** Natalie M. Meléndez-Vázquez, Candelaria Gomez-Manzano, Filipa Godoy-Vitorino

**Affiliations:** 1 Department of Microbiology and Medical Zoology, University of Puerto Rico-Medical Sciences Campus, San Juan, PR 00918, USA; natalie.melendez2@upr.edu; 2 Department of Neuro-Oncology, The University of Texas MD Anderson Cancer Center, Houston, TX 77030, USA; cmanzano@mdanderson.org

**Keywords:** viroimmunotherapy, therapeutic efficacy, gut microbiome, glioblastoma, combinatory therapies

## Abstract

Glioblastoma (GBM) is the most prevalent malignant brain tumor. Current standard-of-care treatments offer limited benefits for patient survival. Virotherapy is emerging as a novel strategy to use oncolytic viruses (OVs) for the treatment of GBM. These engineered and non-engineered viruses infect and lyse cancer cells, causing tumor destruction without harming healthy cells. Recent advances in genetic modifications to OVs have helped improve their targeting capabilities and introduce therapeutic genes, broadening the therapeutic window and minimizing potential side effects. The efficacy of oncolytic virotherapy can be enhanced by combining it with other treatments such as immunotherapy, chemotherapy, or radiation. Recent studies suggest that manipulating the gut microbiome to enhance immune responses helps improve the therapeutic efficacy of the OVs. This narrative review intends to explore OVs and their role against solid tumors, especially GBM while emphasizing the latest technologies used to enhance and improve its therapeutic and clinical responses.

## 1. Introduction

Glioblastoma (GBM) is the most common primary malignant brain tumor and one of the most invasive cancers worldwide. Current therapies against GBM, including surgical resection, chemotherapy, and radiation, have proven to be relatively ineffective, resulting in a median survival of 15 months post-diagnosis [1,2,3] and a 5-year survival rate of 6.8% [3]. Treatment advances against this solid tumor include several types of immunotherapies and targeted therapies. Among these, immune checkpoint inhibitors (ICIs) have proven to be quite unsuccessful in patients with GBM [4,5].

To target the poor survival prognosis associated with malignant gliomas, the development of new therapies is imperative. To tackle this problem, a special type of immunotherapy known as oncolytic viral therapy has shown promising results in preclinical and clinical studies [6]. Advances in the oncolytic viral therapy field have led to US Food and Drug Administration (FDA) approval of talimogene laherparepvec (T-VEC), a modified herpes simplex virus (HSV) type 1 with cancer selectivity, to treat another type of solid tumor, metastatic melanoma [7]. Although oncolytic viruses (OVs) are promising bio-therapeutic agents [8], an important challenge arises with their efficacy due to their high immunogenicity leading to rapid clearance [9]. This paradigm shift has led to the transition from monotherapy to combinatorial therapies, where some enhancement in efficacy and overall survival has been observed when combining OVs with chemotherapy, ICIs, and targeted therapy [10].

Several biological factors may contribute to determining a patient’s responsiveness to cancer therapies. Given the expansion of human microbiome studies in the past 12 years, we now know that the gut microbiota is associated with a myriad of diseases. The integration of the human gut microbiota into the hallmarks of cancer underscores its pivotal role in shaping overall human health [11]. It is, therefore, an important biological factor to consider when proposing new anti-cancer therapeutics. In particular, a close relationship between the gut microbiota and immunotherapy efficacy has been described [12,13,14,15]. The bacterial taxa *Bifidobacterium* has been associated in preclinical [13] and clinical [16] settings with an anti-PD-L1 treatment response. Specifically, a higher gut diversity and an increase in *Ruminococcaceae* and *Faecalibacterium* have been associated with anti-PD-L1 therapy response in melanoma patients [17]. In addition, *Bifidobacterium* supplementation has been assessed regarding the response to immunotherapy [13,18,19,20,21] and oncolytic virotherapy [22]. In the context of oncolytic adenoviruses, *Bifidobacterium* supplementation has also been associated with therapeutic response in a melanoma preclinical model [22]. Some other studies have also found the role of the mycobiota (fungal communities) in cancer therapy response [23,24]. Antibiotic-induced bacterial depletion in an animal model led to overgrowth of commensal fungi, thereby impairing response to radiotherapy [23]. Likewise, suppression of tumor growth and metastasis has been observed with the yeast *Saccharomyces cerevisiae* on in vitro assays and animal models from colon cancer and melanoma [25,26]. This narrative review explores the potential association between gut microbial communities and oncolytic viral therapy efficacy, while also assessing modulation strategies that may enhance this synergistic relationship.

## 2. Malignant Gliomas: The Problem and Current Therapeutic Approaches

### 2.1. Epidemiology of Glioblastoma

GBM, also known as glioblastoma, IDH-wildtype, is a diffuse astrocytic glioma with no mutation in the isocitrate dehydrogenase 1 (IDH1) or IDH2 genes [27]. Although little is known about its etiology, there are some risk factors associated with its development which include (1) increasing age, (2) ionizing radiation therapy, (3) individuals with a rare genetic syndrome (e.g., Turcot syndrome, Lynch syndrome, and Li-Fraumeni syndrome), and (4) people with familial history for brain tumors may develop the same kind of tumors [28,29]. The clinical presentation will vary according to tumor location; however, the most predominant symptoms are cognitive impairment, seizures, persistent headaches, dysphagia, drowsiness, and confusion [30].

GBM is the most common primary malignant brain tumor and has a worldwide incidence of 1.6%, being more predominant in males than females [3]. These brain tumors are associated with a median survival of 15 months post-diagnosis in spite of the standard of care, which consists of surgical resection, chemotherapy, and radiotherapy [1,2,31]. Recurrence is virtually inevitable for this cancer, highlighting the poor survival prognosis of patients, where only 6.8% survive more than 5 years [3]. In the United States (USA), GBM has an incidence rate of 3.27 per 100,000 population, accounting for 50.9% of all central nervous system (CNS) malignant tumors [3]. Recently, more studies have delved into the applications of different immunotherapies. In the following sections, we discuss in more detail the treatment options currently available for GBM.

### 2.2. Treatment Options for GBM

Surgical resection is the initial approach of standardized care to tackle GBM [2]. Its goal is to effectively eliminate as much of the tumor as possible while preserving neurological function [32]. Evidence underscores the association between the maximization of surgical resection and longer life expectancy for low- and high-grade gliomas [33]. Nonetheless, it is not a stand-alone therapy as surgery cannot completely eradicate GBM, and recurrence occurs in approximately 80% of the patients [34]. Radiation therapy (RT) is typically followed by resection, optimally within 3–5 weeks after surgery [35], enhancing local control while minimizing the risk of neurotoxicity [32]. It also decreases symptom severity while improving patient social functioning [36,37,38]. In an effort to improve the overall survival of GBM patients, several chemotherapeutic drugs have been developed, including the most used temozolomide (TMZ), bevacizumab, lomustine, and carmustine [39]. Since FDA approval in 2005, the alkylating agent TMZ has been the current standard of care for newly diagnosed GBM. Even with positive outcomes, given the mutagenic and heterogenic nature of GBM, TMZ resistance is acquired by the tumor which limits the efficacy of the treatment [40,41]. Moreover, with the introduction of the Stupp regimen, which combines TMZ with RT, an increase in overall survival has been achieved [1,42]. However, the 5-year survival rate still shows no apparent enhancement [43]. In the case of bevacizumab, an anti-angiogenic chemotherapeutic agent, it has become a popular second-line treatment, although it has provided limited benefits, improving only progression-free survival (PFS) [44,45,46,47]. Lastly, both lomustine and carmustine are non-specific alkylating agents that cause DNA/RNA crosslinking and are commonly used for high-grade malignant gliomas [39]. These non-tumor-specific therapies lead to several adverse events such as nausea, vomiting, fatigue, body pain, and bleeding gums [34].

Due to the limited benefits offered by the previously mentioned therapies, clinical efforts have shifted towards advancing immunotherapies against solid tumors. Immunotherapy approaches can be divided into active and passive immunotherapy. The two strategies under active immunotherapy that have shown promising progress against GBM are peptide-based therapy [48] and cell-based therapy, specifically with dendritic cell (DC)-based vaccines mediated through immunogenic cell death [49,50,51]. These vaccine therapies targeting tumor-associated antigens and tumor-specific antigens have been tested against GBM in phase I, II, and III clinical trials [52,53,54]. On the other hand, passive immunotherapy showcasing potential avenues for enhancing GBM prognosis include monoclonal antibodies, such as ICIs [55,56], and adaptive immunity through chimeric antigen receptor (CAR) T-cell therapy. Specifically, CAR T-cell therapy targets tumor surface molecules such as epidermal growth factor receptor variant III (EGFR variant III) [57], interleukin 13 receptor subunit alpha 2 (IL13Rα2) [58], and human epidermal growth factor receptor 2 (HER2) [59]. A case report from a phase I clinical trial with CAR T-cell therapy targeting IL13Rα2 observed tumor regression in a recurrent multifocal GBM patient [60]. The final results of this clinical trial showed disease stability in 50% of the patients, including two partial responses and one complete response with an increase in inflammatory cytokines such as IFNγ, CXCL9, and CXCL10 [58]. Another phase I clinical trial that is currently undergoing published preliminary results from three recurrent GBM patients being treated with CARv3-TEAM-E T cells; these are CAR T cells that target EGFR variant III and the wild-type EGFR protein through the secretion of a T-cell–engaging antibody molecule (TEAM) [61]. Even though tumor regression in this subset of patients was rapid, after one sole dose, and only days after treatment, the response was limited as tumors tended to reappear [61]. Immune checkpoint blockade is a modulatory immunotherapeutic approach that encompasses anti-PD1, anti-PD-L1, and anti-CTLA-4. These ICIs target specific tumor surface antigens, reducing off-target toxicity when compared to traditional chemotherapy [56]. Preclinical and clinical studies [62,63,64] have demonstrated substantial positive outcomes, and a notable surge of FDA approvals for cancer immunotherapies against several malignancies has been occurring for years [65]. However, since the efficacy of ICIs is restricted to only a subset of patients, with 60–70% remaining unaffected, this highlights the need for combinatorial therapies [66,67]. In the GBM context, several studies have been conducted to better understand the benefits of ICIs. Both in vitro and in vivo GBM assays showed that PD-1 blockade monotherapy induced long-term response, and combination therapy with either TMZ or RT underscored the enhanced efficacy [68,69]. While preclinical models show promise, clinical trials do not showcase the same efficacy [4,70,71,72,73]. Still, there are currently a few phase II clinical trials ongoing, including a study evaluating pembrolizumab, another anti-PD1 drug, in combination with RT in patients with recurrent GBM (Clinical Trial ID: NCT04977375). Although CTLA-4 and PD/PD-L1 are the most studied ICIs, research is also exploring other pathways targeting lymphocyte activation gene-3 (LAG-3) and T-cell immunoglobulin and mucin-3 (TIM-3) [74,75].

GBM is described as a cold tumor due to several factors that contribute to immune system evasion (Figure 1). One of these factors is the high expression of indoleamine-2,3-dioxygenase (IDO), a tryptophan-degrading enzyme that converts tryptophan to kynurenines [76]. This metabolic shift in the ratio of tryptophan and kynurenines results in immunosuppression through the recruitment of regulatory T cells (Tregs) as well as apoptosis of T-cells and antigen-presenting dendritic cells (DCs) [77,78,79]. Downregulation of IDO, through IDO inhibitors such as indoximod, has shown promising enhancement in the survival prognosis of GBM patients [80,81,82,83]. Epacadostat, another IDO inhibitor, has been evaluated in patients with other solid tumors, yielding inconsistent outcomes across studies [84,85]. It is currently being tested in a phase II clinical trial for recurrent GBM (Clinical Trial ID: NCT03532295). Despite these advancements, the limited success in improving GBM survival remains a persistent challenge. Thus, to address the poor survival prognosis of malignant gliomas, the development of novel therapies is imperative.

## 3. Oncolytic Viruses in the Fight Against Malignant Gliomas

### 3.1. What Are Oncolytic Viruses?

To tackle the poor survival prognosis of malignant gliomas, a special type of immunotherapy known as oncolytic viral therapy has been under the spotlight, showing promising results in preclinical and clinical studies [86,87,88,89,90,91,92]. OVs can be lab-engineered and non-engineered viruses that potentiate antitumor immunity through direct and indirect mechanisms. They selectively replicate within tumor cells, resulting in the destruction of the cancerous tissue [93]. This leads to the liberation of more viral particles, which continue the infection of adjacent tumor cells and the release of tumor- and viral-associated antigens that are presented to T cells by neighboring DCs [94]. They also release cytokines such as type I interferons (IFNs), tumor necrosis factor-α (TNFα), and interleukin-12 (IL-12), which promote antigen-presenting cell (APC) maturation [93]. Thus, activating and migrating tumor- and virus-specific CD8^+^ T cells to the tumor, where chemokines also enhance immune cell infiltration, leads to immune-mediated tumor destruction [95]. Therefore, an immune response is mounted against both the tumor and the virus, highlighting the limited time frame of direct oncolysis the therapy executes. This TME remodeling facilitates the transformation of immunogenically cold tumors, like GBM, into hot tumors; thus, enhancing the therapy response rate [96].

Several viruses, from DNA and RNA genetic backbone, have been proposed as potential OVs including adenoviruses [97], poliovirus [98], poxviruses [99], HSV-1 [97], coxsackieviruses [100], reovirus [101,102], measles virus [103], and Newcastle disease virus [104,105]. Many are currently being tested in both preclinical and clinical studies against solid tumors as monotherapy or in combination with other therapies [101,106]. Oncolytic virotherapy has been extensively studied for metastatic melanoma, resulting in FDA approval of the first OV to treat this solid tumor in 2015—a modified HSV-1 with cancer-selectivity named T-VEC [7].

### 3.2. Viroimmunotherapy Advancements in Gliomas

These replication-competent viruses are also being extensively tested against GBM and show encouraging results [90,91,92,107], being the most common adenoviruses [95], poliovirus [98], and HSV-1 [108]. Among the adenoviruses, Delta-24-RGD (DNX-2401) emerges as a pivotal therapeutic in several clinical trials. DNX-2401 is a tumor-selective, replication-competent oncolytic adenovirus, encompassing a mutation in the retinoblastoma protein-binding region of the early region 1A (E1A) and the insertion of the peptide motif RGD-4C in the HI-loop of the fiber to enhance infectivity [109]. Particularly, the oncolytic adenovirus Delta-24-RGD induced complete tumor regression in 20% of patients with recurrent GBM in a phase I clinical trial [90]. Additional clinical trials with Delta-24-RGD against adult and pediatric patients with malignant gliomas or diffuse intrinsic pontine gliomas (DIPGs) have shown encouraging results (Clinical Trial ID: NCT02798406 and NCT03178032) [91,92]. Specifically, 56.2% of patients showed either stable disease or clinical responses with a combination of Delta-24-RGD and pembrolizumab, with an extended survival of up to 60 months in a subset of patients [92]. Similarly, in the clinical trial using Delta-24-RGD with standard-of-care RT in pediatric patients with a new diagnosis of DIPG, a reduction in tumor size was reported in 9 patients, partial or stable responses in 11 of the 12 patients, and a median survival of 17.8 months [91]. To improve the efficacy of Delta-24-RGD, a new generation of adenovirus, named Delta-24-RGDOX, was developed to express the immune costimulatory OX40 ligand (OX40L), which enhances tumor-specific T cell activation as well as the antigen-presenting capabilities of tumor cells [110]. Similarly, preclinical studies with Delta-24-RGDOX (clinically known as DNX-2440) have demonstrated a more robust anti-tumor T cell response than Delta-24-RGD in GBM and metastatic melanoma mice models [111,112].

Another promising candidate is an oncolytic polio-rhinovirus recombinant agent named PVS-RIPO. To decrease the neuropathogenicity of the poliovirus, its internal ribosomal entry site (IRES) was exchanged with that of the human rhinovirus type 2 [113]. This allowed for viral replication within GBM cells as the human poliovirus receptor, CD155, is commonly expressed in glioma tumor cells [114,115]. A phase I clinical trial of PVS-RIPO in patients with recurrent grade IV malignant glioma resulted in a survival rate of 24–36 months in 21% of patients, with two surviving more than 69 months (Clinical Trial ID: NCT01491893) [116]. It has also been tested in pediatric high-grade gliomas for safety and toxicity, showcasing a median survival of 4.1 months and one patient surviving beyond 22 months (Clinical Trial ID: NCT03043391) [117]. The University of California at San Francisco is currently undergoing a phase II clinical trial with PVS-RIPO against recurrent malignant glioma to assess safety and efficacy (Clinical Trial ID: NCT02986178). Moreover, an active clinical study, which is still awaiting the start of recruitment, involves the combination of PVS-RIPO with pembrolizumab to treat recurrent GBM patients (Clinical Trial ID: NCT04479241).

HSV-based therapies are some of the most studied for OV development due to three main reasons: (1) the small-sized genomes, which make it easy to manipulate, (2) modified surface glycoproteins that can target cell receptors, and (3) because viral replication is easily manageable with specific anti-viral drugs [108]. The most known oncolytic HSV is T-VEC, the first FDA-approved OV against inoperable melanoma [7]. This paved the way for the development of more robust and safer oncolytic HSVs against solid tumors, including GBM. Teserpaturev, also known as HSV-1 G47Δ, has three main modifications: (1) the deletion of the *γ34.5* gene, which allows for a decrease in viral pathogenicity; (2) an insertion on the *UL39* gene which promotes viral replication on dividing cells; and (3) the deletion of the *α47* gene and *US11* promoter region, enhancing viral replication [118,119,120]. In a phase I/II clinical study with HSV-1 G47Δ against progressive glioma, the median overall survival from the initial diagnosis was 30.5 months and 7.3 months from the last dose of the therapy, where 3 out of 13 patients survived more than 46 months [121]. Further advancement from a phase II clinical trial of 19 patients with GBM found a one-year survival rate of 84.2% and a median overall survival of 20.2 months after HSV-1 G47Δ treatment, where three patients survived for more than 3 years [122]. These encouraging results led the regulatory agency of Japan to grant conditional and time-limited approval to teserpaturev (G47∆; Delytact) for the treatment of patients with malignant glioma. rQNestin34.5v.2, also known as rQNestin, is another oncolytic HSV-1 that is currently in the recruiting stage of the phase I clinical trial for recurrent glioma (Clinical Trial ID: NCT03152318). M032-HSV-1 is another oncolytic virus modified to express the subunits p35 and p40 of IL-12, stimulating an anti-angiogenic effect [123,124]. Currently, there are two ongoing phase I clinical trials to test the efficacy and safety of this therapy, both in children and adults, against brain tumors (Clinical Trial ID: NCT02457845 and NCT02062827, respectively). In June 2024, in vitro and in vivo studies assessed the safety and efficacy of a new generation of the oncolytic HSV-1 C5252, armed with anti-PD-1 and IL-12 [125]. Researchers found a promising therapeutic prospect against GBM [125], highlighting the need for further clinical translational studies.

One of the latest oncolytic viral candidates against GBM is the Newcastle disease virus (NDV). This avian paramyxovirus is non-pathogenic to humans and its oncolytic potential comes naturally from its preference to replicate within cancerous cells [126]. A preclinical study with an orthotopic syngeneic murine GL261 GBM model treated with NDV showcased long-term survival in 50% of the animals through the induction of immunogenic cell death [127]. Another study performed in vitro and in vivo GBM models to assess the recombinant NDV (rNDV) expressing the human phosphatase and tensin homolog (PTEN) gene (rNDV-PTEN) [128]. Viral treatment with rNDV-PTEN to the GBM cell line U87-MG showed a reduction in cell proliferation and migration as well as induction of apoptosis [128]. Similar results were also seen in the orthotopic GBM murine model, where viral therapy reduced tumor size and enhanced survival [128]. An athymic nude GBM mice model treated with the recombinant NDV Anhinga strain, carrying the tumor necrosis factor-related apoptosis-inducing ligand (TRAIL), achieved a significant reduction in tumor growth when compared to controls [129]. Furthermore, in vitro studies have assessed the potential of combination therapies. Specifically, TMZ-loaded polylactic-co-glycolic acid (PLGA) nanoparticles alongside NDV therapy against the GBM cell line AMGM5 revealed synergistic enhancement of the anti-cancer immune response [130]. Similar findings were also observed with the NDV LaSota strain in combination with TMZ [131]. Although preclinical findings have been promising with NDV against GBM, clinical studies have been limited [132,133].

Although OVs are promising bio-therapeutic agents [8], tumor immune heterogeneity, fast clearance by the immune system [9], and the immunosuppressive state of the TME [134,135] affect therapy efficacy. Therefore, there is a window of opportunity to improve this therapy by combining OVs with other strategies such as chemotherapy, ICIs, targeted therapies, and gut microbiota modulation [10].

## 4. Potential of Gut Microbiome Modulation to Enhance Viroimmunotherapy

### 4.1. Role of the Gut Microbiota in Cancer

The gut microbiome is essential to human health and an important immunomodulatory agent. It is involved in physiological processes that impact nutrition uptake, immune system development and regulation, pathogen protection, maintenance of gut integrity, and anti-inflammatory properties [136]. The impact of modernization through a low-fiber diet with high-carb and sugar intake, antibiotic abuse, sanitation, and chemical antimicrobials has led to, in some cases, permanent dysbiosis—an imbalance of these microbial communities and major bacterial extinctions [137]. During the last decade, the gut microbiome has been extensively studied and its association with disease development and therapeutic efficacy has started to be identified [137,138]. Recent advancements have pinpointed the importance of the human gut microbiota, resulting in its integration into the hallmarks of cancer [11]. New technologies are being developed to help us decipher the role of the microbiota in cancer. For instance, the development of a 3D quantitative in situ intratumoral microbiota imaging strategy facilitates the detection of bacterial lipopolysaccharide (LPS) inside human glioma tissue [139]. These findings help provide insight into the intrinsic communication occurring between microbial populations and the TME.

Most research on the associations between gut microbiota and cancer has prioritized the bacterial component, with relatively few studies examining fungi and other gut commensals. One of the most studied bacteria in association with cancer is *Helicobacter pylori*. It is the only bacteria in the International Agency for Research on Cancer (IARC) list of carcinogens [140]. Even though *H. pylori* is an indigenous stomach bacterium that evolved with humans and lowered its prevalence due to urbanized lifestyles [141,142], studies have found a causative role in cancer development [143]. Notably, the eradication of *H. pylori* has provided a risk reduction in gastric cancer [144]. Other bacteria, notably *Fusobacterium nucleatum*, have been associated with colorectal cancer and have been identified in rectal biopsies [145]. Furthermore, *F. nucleatum* can promote liver metastasis, underscoring the important role of the microbiome in cancer progression [146]. In a like manner, the gut microbiome may be involved with glioma formation and regulation through the bidirectional communication that exists between the gut–brain axis. GBM mouse models have shown how tumor presence can induce shifts in the gut microbiota, including an increase in the Firmicutes/Bacteroidetes ratio—a marker for gut dysbiosis [147,148]. Researchers also evaluated GBM growth according to the gut microbiome, finding that the tumor development rate in mice was lower in those that received antibiotic treatment followed by a fecal matter transplant (FMT) compared to the controls [148]. In animals that received only antibiotics, FOXP3 levels in the brain were downregulated due to gut microbial dysbiosis, leading to glioma growth [148]. These results highlight the necessity for balanced gut microbial dynamics on GBM progression. Two Mendelian randomization studies also uncovered a potential protective role of the family *Ruminococcaceae* against GBM development, highlighting a higher abundance of these bacteria is associated with reduced risk [149,150].

In terms of the gut mycobiota, very little is known about their role in GBM. One of the biggest studies to characterize the cancer mycobiome tested over 17,000 patient samples across 35 cancer types to define specific fungal signatures per each cancer [151]. Interestingly, they discovered most identified fungal species resided intracellularly, and for GBM the detected taxa were *Malasseziomycetes*, *Saccharomycetes*, and *Diothideomycetes* [151]. One of the few studies on gut fungal communities exploring the changes in colorectal adenomas revealed a higher abundance of *Phoma* and *Candida* compared to adjacent non-adenoma tissue [152]. Specifically, *Candida albicans* has been associated with a more immunosuppressive state through an increase of PD-1^+^CD8^+^ T cells [23] and inducing neutrophilic myeloid-derived suppressor cells [153]. Other opportunistic fungal pathogens, such as *Malassezia globosa*, have been found to promote pancreatic oncogenesis via complement cascade activation and IL-33 secretion [154,155], as well as shorten overall survival in breast cancer [151]. Moreover, tumor growth and metastasis inhibition have been seen in both in vitro and preclinical models with the yeast *Saccharomyces cerevisiae* [25,26].

In addition to bacterial and fungal taxa, microbial metabolites influence the host metabolism and immune system in both direct and indirect mechanisms [156,157,158,159,160,161]. Colibactin, a potent genotoxin produced by *Escherichia coli* and other members of the *Enterobacteriaceae* family, is one of the major contributors to colorectal cancer development [162]. Another metabolite is short-chain fatty acids (SCFAs), which are formed from carbohydrate fermentation by gut commensals such as *Lactobacillus* and *Bifidobacterium* [163]. Among SCFAs, the most represented are acetate, propionate, and butyrate. These organic molecules can circulate through the body and regulate microglia maturation and function [164]. One of the most studied microbial metabolites in relation to cancer therapy response is butyrate. This SCFA has been associated with tumor suppression and clearance in different cancers via the regulation of apoptosis, autophagy, as well as onco- and tumor-suppressor genes [165,166,167,168]. Butyrate has also been associated with CD8^+^ T cell function modulation and antitumoral properties [157,159]. Dietary tryptophan metabolism is also regulated by gut bacterial communities, which leads to the production of aryl hydrocarbon receptor (AHR) agonists [169]. The AHR is a ligand-activated transcription factor involved in the regulation of several physiological processes including the immune system. As mentioned previously, GBM produces high levels of kynurenines, which cause an immunosuppressive state. One of the mechanisms by which kynurenines achieve this is through the activation of AHR on tumor-associated macrophages (TAMs), promoting antitumoral immune dysfunction [170]. Therefore, gut microbial communities can help disrupt this immunosuppression with the production of AHR agonists. Moreover, in the context of fungal metabolites, in vitro assays have discovered several *Aspergillus*, *Penicillium*, and *Talaromyces*-derived metabolites displaying cytotoxic activity against several cancer cell lines, including GBM [171]. These filamentous fungi are producers of anticancer metabolites belonging to diverse compound families such as alkaloids and polyketides [171]. Similarly, the anti-cancer effect on in vitro studies against GBM cells has been tested with edible mushrooms [172]. Specifically, when evaluating four different fungal extracts, *Coprinus comatus* and *Lactarius delicious* showcased the most cytotoxic activity mediated in a dose-dependent manner against the human GBM cell lines U87MG and LN-18 [172].

Overall, these studies suggest a potential impact of the bacteriome and mycobiome on the host immune response, highlighting their crucial role in cancer biology. It also underscores the delicate balance and co-existence between fungi and bacteria. This emphasizes the need for more in-depth research to continue understanding their synergistic relationship, as they also provide potential targets for therapeutics.

### 4.2. Gut Microbiome Association with Different Cancer Treatment Responses

Several studies have exhibited the close relationship between gut bacterial and fungal communities with cancer therapy response [12,13,14,15,23,24,25,26]. Antibiotic-driven bacterial depletion in preclinical solid tumor models resulted in the overgrowth of commensal fungi, including *Saccharomyces* and *Candida*, which hindered RT response [23]. In addition, in the breast cancer preclinical model, the presence of Dectin-1 in the tumor tissue recognizing the β-glucan of the fungal cell wall after RT supports the hypothesis that through this ligand-receptor interaction, the response rate of RT is modulated [23]. These findings showcase the importance of both bacterial and fungal components of the gut microbiome in regulating gut homeostasis and anti-cancer immunity after treatment. On the other hand, phase II clinical trials have shown that the systemic administration of β-glucan, one of the most abundant polysaccharides in the fungal cell wall, has resulted in enhanced cancer monotherapy treatment such as monoclonal antibodies [173,174]. For chemotherapeutic drugs, the gut microbiome has also been linked to modulating its efficacy. Cyclophosphamide (CTX), a common alkylating agent, causes microbial dysbiosis with a reduction of Lactobacilli and Enterococci in melanoma and sarcoma-bearing animals [175]. This microbial disruption affected the response of “pathogenic” Th17 (pTh17) cells, which consequently drove CTX resistance [175]. Another study with the chemo drug gemcitabine found that intratumoral Gammaproteobacteria, mainly from the *Enterobacteriaceae* and *Pseudomonadaceae* families, conferred drug resistance by its metabolization, which was dependent on the presence of a long isoform of the bacterial enzyme cytidine deaminase (CDD_L_) [176]. A study with C57BL/6 mice implanted with a GL261 GBM tumor highlighted that the induction of *Akkermansia* and *Bifidobacterium* may contribute to the anti-tumor effect of the chemo drug TMZ [177].

Baseline stool samples from 42 metastatic melanoma patients, prior to immunotherapy initiation, unveiled an association between the gut microbiome and clinical response [12]. PD-1 and CTLA-4 blockade responders (16/42; 38%) revealed higher levels of *Bifidobacterium longum, Collinsella aerofaciens,* and *Enterococcus faecium*, while non-responders (26/42; 62%) exhibited more abundance of *Ruminococcus obeum* and *Roseburia intestinalis* [12]. A study on melanoma-bearing mice treated with anti-PD-L1 also found an association between the gut commensal bacteria *Bifidobacterium* and anti-tumor T-cell response [13]. When evaluating the bacterial communities of anti-PD-1 therapy responding patients (30/43; 70%), researchers found a higher gut microbiome diversity associated with significantly increased PFS [17]. Fecal sample assessment between responders and non-responders to anti-PD-1 identified enrichment of *Ruminococcaceae* and *Faecalibacterium* in responders, while *Bacteroides thetaiotaomicron, Escherichia coli*, and *Anaerotruncus colihominis* in non-responders [17]. Moreover, the use of taxonomic level categorization to assess therapy response uncovered that those patients with a high abundance of *Faecalibacterium* had prolonged PFS compared to those with a low abundance [17]. On the other hand, patients with high levels of *Bacteroidales* were associated with reduced PFS compared to those with low levels [17]. Similar findings were also seen with anti-CTLA-4, where patients’ baseline gut microbiota that had enriched *Faecalibacterium* had longer PFS compared to those with higher baseline levels of *Bacteroidales* [178]. Furthermore, immune response analysis showcased those patients with higher levels of *Faecalibacterium* had elevated density of immune cells, including more effector CD4^+^ and CD8^+^ T cells, and markers of antigen processing and presentation [17]. This is contrary to patients with a higher abundance of *Bacteroidales* who had Tregs and myeloid-derived suppressor cells (MDSCs), compromising anti-tumoral immune response [17]. *Faecalibacterium* has been associated with positive responses to immune checkpoint inhibitors across multiple cancer types, improving dysbiosis of inflammatory bowel disease [179] and suggesting its potential as a new probiotic in many cancer treatments [180]. Similarly, previous studies have focused on the anti-inflammatory role of *Akkermansia muciniphila* in the colon [181] and its association with better response to PD-1 blockade therapy [14,182]. Patients treated with CAR-T cell therapy who had a higher abundance of *Akkermansia muciniphila* have also been associated with increased PFS, whereas a larger abundance of *Bacteroides* was linked to lower PFS [183]. It is currently observed that immunotherapy response varies according to *Akkermansia* levels, where absence or overabundance can result in treatment unresponsiveness [182]. For anti-CTLA-4 therapy, broad-spectrum antibiotic administration has compromised the anti-tumoral effects of the treatment [15]. Likewise, solid tumor preclinical models administered an antibiotic cocktail of vancomycin, imipenem, and neomycin, showed impairment of CpG-oligonucleotide immunotherapy, which affected tumor growth, survival, TNF, and cytokine production [184]. Moreover, antibiotic exposure prior to starting immunotherapy has been associated with reduced PFS and overall survival [183]. An assessment of fungal communities across multiple geographical locations and cancer types revealed potential biomarkers of ICI response [24]. A machine learning predictive model, considering datasets across four human cohorts, identified 20 fungal species enriched in responders and 6 in non-responders to anti-PD-1 [24]. An evaluation of the multi-kingdom network identified *Schizosaccharomyces octosporus* as one of the most prominent potential biomarkers for anti-PD-1 response and was found to have an excellent predictive performance with an average receiver operating characteristic (ROC) of 0.87 [24].

Studies regarding gut microbiome association with oncolytic viral therapy efficacy have been limited. Previously, a study found a higher abundance of *Bifidobacterium* and *Akkermansia* associated with response to the oncolytic adenovirus Delta-24-RGDOX along the gut–glioma axis [147]. In this preclinical GBM model, responders to the OV had similar richness and diversity to that of naive animals when compared to untreated mice [147]. We also assessed the role CD4^+^ T cells had on gut microbiota modulation associated with Delta-24-RGDOX efficacy. CD4^+^ T cell depletion resulted in less survival and a higher Firmicutes/Bacteroidetes ratio compared to the OV-treated group with functional CD4^+^ T cells [147]. In addition, we observed a reduction in *Bifidobacterium* as well as other anti-inflammatory taxa such as *Lactobacillus*, *Ruminococcaceae*, and *Lachnospiraceae* due to the depletion [147]. Another study with melanoma-bearing animals undergoing vancomycin administration and oncolytic viral therapy with Ad5D24-CpG showcased faster tumor growth and reduced IFN-γ-producing CD8^+^ T cells compared to the OV-treated animals [22]. Interestingly, melanoma progression was very similar between the combination therapy group (OV and antibiotic) when compared with the mice group administered only the antibiotic, highlighting the use of antibiotics affects viroimmunotherapy efficacy [22]. Although these findings are encouraging, further studies are needed to assess the intrinsic communication that exists between gut microbial communities, GBM, and treatment efficacy.

### 4.3. Strategies for Gut Microbiome Modulation to Enhance Cancer Therapy Response

Studies have evaluated strategies to modulate the gut microbiome to improve response to immunotherapy [21,22,185]. Probiotics, as defined by the International Scientific Association for Probiotics and Prebiotics (ISAPP), are “live microorganisms that, when administered in adequate amounts, confer a health benefit on the host” [186]. These microorganisms, which are typically bacteria but can also include yeasts, are found naturally on fermented foods such as kimchi, kombucha, miso, sauerkraut, and kefir [187]. However, probiotics can also be found commercially with one or more specific strains depicted as “good bacteria” such as *Lactobacillus* and *Bifidobacterium*. As seen previously, *Bifidobacterium* is one of the key bacterial taxa of interest for enhancing cancer therapy response. Therefore, one of the strategies for gut microbial modulation is oral supplementation with *Bifidobacterium* spp., which has improved tumor control and enhanced PD-L1 blockade therapy through CD8^+^ T cell priming and accumulation in the TME [13]. When tested on CD8^+^ T cell-depleted mice, the therapeutic effect of *Bifidobacterium* supplementation, specifically of *Bifidobacterium breve* and *Bifidobacterium longum*, was hindered [13]. In addition, studies inactivating *Bifidobacterium* with heat found the probiotic effects hampered, suggesting the need for live bacteria to achieve the desired anti-tumoral effect [13]. Another study with oral supplementation with several strains of *Bifidobacterium bifidum* showed a reduction in tumor burden with anti-PD-1 therapy and the chemotherapeutic agent oxaliplatin by enhancing anti-tumoral immune response [21]. Interestingly, this enhancement of PD-1 blockade was attained only with a specific subset of strains of *B. bifidum* (*B. bif*_K57, *B. bif*_K18, and *B. bif*_M31), observing an increase in CD4^+^, CD8^+^, and NK cells as well as an increase in the cell ratio of effector CD8^+^ T cells/Tregs [21]. In the case of oxaliplatin, while several *B. bifidum* strains decreased tumor growth, only two strains (*B. bif*_K57 and *B. bif*_K18) worked synergistically with the chemotherapy drug [21]. Immune cell profiling for the combination of oxaliplatin and *B. bifidum* strains showed an increase in effector CD8^+^ T cells and the cell ratio of effector CD8^+^ T cells/Tregs [21]. Probiotic supplementation with *Bifidobacterium* sp. has also resulted in a reduction in melanoma progression and tumor-infiltrating Tregs in a preclinical model treated with the oncolytic adenovirus AD5D24-CpG [22]. The reduction in Tregs was even more significant in the animals only administered the probiotic [22]. The peptidome of *Bifidobacterium* and melanoma were compared, and after careful curation, 10 peptides were identified for *Bifidobacterium* and 14 for melanoma [22]. Interestingly, molecular mimicry was observed between epitopes derived from *Bifidobacterium* and melanoma with in vitro assays and preclinical models, suggesting a possible cross-reactive T cell activation mechanism by which the microbiome modulates viroimmunotherapy response [22]. Given the promising results of probiotic administration in cancer therapy response, clinical trials assessing the potential translational application of gut microbiome therapeutics have been on the rise. Currently, the probiotic Probio-M9, containing *Lactobacillus rhamnosus*, is being evaluated as a potential enhancer of PD-1 blockade against liver cancer (Clinical Trial ID: NCT05032014). Recently, a phase I clinical trial was completed that assessed the probiotic CBM588 (*Clostridium butyricum*) in regard to anti-PD-1 and anti-CTLA-4 efficacy against advanced kidney cancer (Clinical Trial ID: NCT03829111).

Nutrition is one of the most commonly known modifiers of the gut microbiota. Specific nutrients acquired from the diet, also known as prebiotics, can modulate the abundance of beneficial bacterial species in the gut. Prebiotics, a term initially introduced in 1995, was described as “a non-digestible food ingredient that beneficially affects the host by selectively stimulating the growth and/or activity of one or a limited number of bacteria in the colon, and thus improves host health” [188]. However, a revision by the ISAPP refined the concept into “a substrate that is selectively utilized by host microorganisms conferring a health benefit” [189]. This dietary fiber acquired from foods such as vegetables, fruit, whole grains, and legumes select for “good bacteria” within the gut. In a study with melanoma patients undergoing an ICI regimen, of which 193 were responders and 100 non-responders, researchers assessed dietary habits and probiotic usage [190]. Prior to the initiation of ICI treatment, patients completed the National Cancer Institute Dietary Screener Questionnaire from which threshold values for fiber intake were assessed as 5 g per day, with low fiber intake to less than 20 g/day, and high fiber intake at or above 20 g/day [190]. Particularly, patients treated with anti-PD-1 who had high fiber intake showed enhanced PFS when compared with patients with low fiber intake [190]. Further preclinical melanoma models undergoing anti-PD-1 and fed a high-fiber diet demonstrated retarded tumor growth when compared to treated animals fed a low-fiber diet [190]. A clinical trial assessed the prebiotic effect of inulin and fructo-oligosaccharide on *Lactobacillus* and *Bifidobacterium* on gynecologic cancer requiring postoperative pelvic RT (Clinical Trial ID: NCT01549782) [191]. Specifically, their results highlighted how RT led to a reduction in *Lactobacillus* and *Bifidobacterium* with the restoration of these bacterial species after prebiotic administration, suggesting a reduction in intestinal side effects caused by RT [191]. Two more clinical studies are assessing the modulatory effect of prebiotics on colorectal cancer, specifically one with soluble corn fiber (Clinical Trial ID: NCT05516641) and another with polyunsaturated fats (PUFAs) (Clinical Trial ID: NCT04869956). Currently, there’s an active phase II clinical trial evaluating the effects of two types of dietary interventions on the clinical response of immunotherapy-treated melanoma patients (Clinical Trial ID: NCT04645680). Overall, these studies open an avenue in terms of baseline knowledge for future dietary interventions to improve cancer treatments, including the efficacy of viroimmunotherapy.

FMTs are a sought-out strategy to potentially restore host gut homeostasis. In 2010, a patient with chronic diarrhea due to an infection from *Clostridium difficile* achieved a successful gut microbiota restoration after an FMT from a healthy donor [192]. Continuous improvement throughout the decade led to the FDA approving the first microbiota-based treatment named REBYOTA [193]. Another recently approved microbiota-based therapy was SER-109, an oral formulation made from bacterial spores, for recurrent *C. difficile* infection [194]. In terms of immunotherapy efficacy, FMTs have shown promising results in combination with ICIs in both preclinical and clinical studies with refractory melanoma and other solid tumors [14,17,185,195,196]. Melanoma-bearing mice that received FMT from patients who responded to anti-PD-1 therapy were more responsive to the same treatment, highlighted by an immune profile of higher CD8^+^ T cells [17]. Similarly, animals that received FMT from anti-PD-1 non-responders also had a poor response to the therapy [17]. A phase I clinical trial for safety assessment showed that patients had strain colonization from their donors and experienced a decrease in “bad” bacteria, observing an objective response rate of 65% [195]. Another phase I clinical trial evaluating the safety and feasibility of FMTs in changing the poor response rate of anti-PD-1 found a clinical response in three patients as well as positive changes in immune cell infiltrates [185]. A similar finding was also seen in another clinical trial with an increase in CD8^+^ T cell activation and a decrease in myeloid cell immunosuppression (Clinical Trial ID: NCT03341143) [197]. FMTs have also been tested in reducing gut-related side effects, such as colitis, caused by ICI therapy. In a case report of a 71-year-old man with gastric adenocarcinoma and PD-1 blockade treatment, the patient continued to experience severe ICI colitis despite all efforts to reduce symptoms and pain [196]. The FDA approved an FMT for compassionate use where only days after the intervention results showed diminished inflammation, bowel movements, and abdominal pain, with no further return of colitis symptoms [196]. These positive outcomes have led to a phase I clinical trial that is currently recruiting genitourinary cancer patients to assess how FMTs can abrogate diarrhea and colitis caused by ICIs (Clinical Trial ID: NCT04038619). Another phase I clinical study assesses FMT potential in reducing toxicity caused by ICI therapy in renal cancer (Clinical Trial ID: NCT04163289). In terms of potentiating anti-cancer therapy response, a phase II clinical trial is assessing the antitumor enhancement of combining FMTs with ICI therapy on non-small cell lung cancer and melanoma (Clinical Trial ID: NCT04951583). Currently, a phase II clinical trial is recruiting patients to evaluate the safety, feasibility, and efficacy of FMTs to ICI non-responders using as donors ICI responders (Clinical Trial ID: NCT05286294). The use of FMTs is therefore a potential strategy to enhance oncolytic virotherapy. An initial study with a colorectal cancer preclinical model found that FMTs enhance oncolytic virus OVV-gp33 efficacy with an increase in CD8^+^ T cells and a decrease in Treg levels [198]. Further studies should be developed to continue expanding the limited knowledge on FMTs and oncolytic viral therapy efficacy.

The mechanisms by which FMTs improve cancer therapy efficacy are still unknown. However, bacteriophages have emerged as an important component of the gut virome [199,200], playing a role in the modulation of therapeutic efficacy [201,202]. Bacteriophages, also known as phages, are prokaryotic viruses that infect only bacterial species. A batch fermentation model tested a 4-phage myovirus cocktail against a *C. difficile* infection, which resulted in complete eradication [203]. Clinical studies have shown how FMT interventions on patients suffering *C. difficile* infection also introduced phages into the gut microbiome [201,202]. Recently, phage applications have ventured into understanding their potential as enhancers of anti-cancer agents. Specifically, filamentous phages (members f1, M13, and fd) are able to cross the blood–brain barrier and enter the central nervous system without inducing toxicity [204]. This allows phages to effectively penetrate and improve drug delivery to the cancerous tissue [204]. For example, the modified vector RGD4C-AAVP-*TNF*, made from the backbone of an adeno-associated virus (AAV) and a M13-derived bacteriophage, was tested on an orthotopic GBM immunodeficient mice model and showcased tumor regression through cellular apoptosis [204]. Moreover, another variant of this phage, named RGD4C-AAVP-*Grp78*, has shown a synergistic effect with the chemo drug TMZ on an orthotopic GBM mice model, resulting in tumor destruction [205]. On another preclinical GBM model, the intranasal administration of filamentous phages inhibited GBM tumor progression mediated partly by the LPS carried on its virion [206]. These findings highlight the potential of phage therapeutics for combination therapies with oncolytic viruses against GBM.

## 5. Future Perspectives of Gut Microbial Modulation in Combination with OVs

The findings discussed earlier have become a setting stone for further inquiry into gut microbial modulation and viroimmunotherapy efficacy. Given the extensive research on the role of gut microbial communities in physiological processes and host immune system development, its potential as an enhancer of therapeutic agents should not be surprising. As seen with ICIs, certain gut microbes (ex. *Bifidobacterium*) and their secondary metabolites (ex. butyrate) can be potential modulators of oncolytic viral therapy response.

Continued advancements in sequencing technologies will yield increasingly comprehensive in-depth sequences for species and gene identification. The integration of metagenomics with metabolomics, transcriptomics, and proteomics will provide a more nuanced understanding of the molecular dynamics within the gut. This approach may uncover a causal link between viroimmunotherapy response and gut microbial communities. Personalized gut microbial modulation will likely improve the immune response of patients undergoing oncolytic virotherapy resulting in prolonged survival while maintaining a protective gut community throughout time (Figure 2). By modulating the gut microbiome, through probiotic supplementation, diet modulation, or FMTs, the immune landscape may be enhanced, allowing for a more robust anti-tumoral immune response. Specifically, biomarker identification is essential for predicting patient responses, enabling a more meticulous determination of the optimal combination therapies for the effective eradication of GBM. More importantly, there are very limited clinical trials focused on the modulation of the gut microbiome to enhance therapy efficacy. Additionally, a combination of tailored therapies including metagenomic data with individualized phage therapies based on a patient’s unique microbiome profile, jointly with probiotics, prebiotics, or immune modulators for a multifaceted approach is also promising.

Further studies are warranted to unravel the mechanisms of FMT, diet modulation, and probiotic supplementation to determine which strategy is ideal for enhancing OV efficacy against GBM. Overall, combining gut microbial modulation with oncolytic viral therapy efficacy presents a frontier for personalized cancer medicine, having the potential to revolutionize patient outcome.

## 6. Conclusions

Combination therapies of OVs and the gut microbiome is an emerging and promising field that warrants further studies. While OVs have enhanced clinical response and extended overall survival in malignant gliomas, a subset of patients still does not respond to therapy. The gut microbiome is an undeniable biological factor that contributes to health and therapy response. Henceforth, future strategies regarding oncolytic viral therapy enhancement should include gut microbiome modulation through probiotic supplementation, metabolic profiling, and FMTs.

## Figures and Tables

**Figure 1:** OV-mediated cold tumor transformation into hot tumor exhibits immunological features that may enhance the response to immunotherapeutic agents against glioblastoma. Created in BioRender. [Laboratory, M. (2024) BioRender.com/m60l030 (accessed on 28 October 2024).]

**Figure 2:** Restoration of the gut microbiota of a non-responsive patient to oncolytic viral therapy from an FMT of a responder donor with an adjuvant diet to improve the establishment of gut commensals and SCFA production. Special emphasis on the antitumoral effects of the restored microbiota on the oncolytic virus. Created in BioRender. Laboratory, M. (2024) BioRender.com/q49i287 (accessed on 28 October 2024).
